The article "3D Printed Guides and Preoperative Planning for Uncemented Stem Anteversion Reconstruction during Hip Arthroplasty: A Pilot Study" was retracted in 2024. Reasons: suspected computer-generated content; unreliable results or conclusions; concerns about the data; concerns about the results or conclusions.

# 3D Printed Guides and Preoperative Planning for Uncemented Stem Anteversion Reconstruction during Hip Arthroplasty: A Pilot Study

**DOI:** 10.1155/2021/6621882

**Published:** 2021-02-19

**Authors:** Yingqi Zhang, Zhitao Rao, Jincheng Zhang, Shijie Li, Shimin Chang, Yeqing Sun

**Affiliations:** ^1^Department of Orthopedic Surgery, Tongji Hospital, Tongji University School of Medicine, Shanghai 200065, China; ^2^Department of Orthopedic Surgery, Yangpu Hospital, Tongji University School of Medicine, Shanghai 200090, China

## Abstract

**Objective:**

To investigate if 3D printed guides and preoperative planning can accurately control femoral stem anteversion.

**Methods:**

A prospective comparative study was carried out from 2018 to 2020, including 53 patients who underwent hip arthroplasty for femoral neck fracture. The target rotation center of the femoral head is determined by three-dimensional planning. In group A, planning was made by 2D templates. In group B, preoperative 3D planning and 3D printed osteotomy/positioning guides were performed. After the operation, 3D model registration was performed to calculate the accuracy of anteversion restoration.

**Results:**

We screened 60 patients and randomized a total of 53 to 2 parallel study arms: 30 patients to the group A (traditional operation) and 23 patients to the group B (3D preoperative planning and 3D printed guide). There were no significant differences in demographic or perioperative data between study groups. The restoration accuracy of group A was 5.42° ± 3.65° and of group B was 2.32° ± 1.89°. The number and rate of abnormal cases was 15 (50%) and 2 (8.7%), respectively. Significant statistical differences were found in angle change, restoration accuracy, and number of abnormal cases.

**Conclusion:**

Three-dimensional preoperative planning and 3D printed guides can improve the accuracy of the restoration of femoral anteversion during hip arthroplasty.

## 1. Introduction

Hip arthroplasty is an extremely successful procedure, which help improving range of motion and decreasing pain and finally improving patients' quality of life [1, 2]. However, mispositioning of the implants can result in premature implant failure requiring revision [1–4]. Although the most common cause of revision surgery was due to cup mispositioning (33%), surgeons should be aware of the variability of the femoral anteversion of uncemented stems [5, 6]. The traditional methods of using preoperative anteroposterior pelvis radiographs for planning and standard surgical instrumentation have shown potential for inaccuracy which varies with surgeon experience. With the development of digital orthopedics, CT-based three-dimensional planning and navigation systems have been introduced to improve the accuracy of prosthesis implantation [7–9]. However, the implantation of the femoral stem is affected by the surgical incision, visual field, and irregular medullary cavity shape of the proximal femur. It is difficult to accurately restore the anteversion, even based on preoperative CT measurement results [6, 10].

3D printed personalized guides have been used in orthopedic surgery in recent years and have achieved good results [11, 12]. Based on a patient's unique bony morphologic features is an improvement over generic instruments by minimizing sources of error from standard surgical instruments that depend on appropriate patient positioning, exposure, and surgeon experience [13–15]. However, there are rare reports in the previous literature about the use of guide to assist the femoral anteversion restoration [6]. Based on the preoperative three-dimensional planning, we developed a femoral osteotomy guide and a stem positioning guide. For hip arthroplasty, it is expected to accurately restore the femoral anteversion.

The article "3D Printed Guides and Preoperative Planning for Uncemented Stem Anteversion Reconstruction during Hip Arthroplasty: A Pilot Study" was retracted in 2024. Reasons: suspected computer-generated content; unreliable results or conclusions; concerns about the data; concerns about the results or conclusions.

## 2. Materials and Methods

This prospective, controlled trial was performed from January of 2018 to January of 2020 at a single large academic institution. This study was approved by our institutional review board, and every patient gave written informed consent to participate.

### 2.1. Patients

Patients scheduled for a primary arthroplasty were approached for the study. Inclusion criteria are as follows: (1) unilateral traumatic femoral neck fracture, (2) primary hip replacement, (3) age > 18 years old at time of surgery, (4) cementless straight stem (Johnson & Johnson/Zimmer Biomet, USA), and (5) able to get a preoperative and postoperative CT scans. Exclusion criteria are as follows: (1) hip joints had abnormalities before this injury and (2) condition deemed by physician to be nonconductive to patient's ability to complete the study. Demographic information collected on all patients was age, gender, and body mass index (BMI).

### 2.2. Three-Dimensional Planning

In all cases, the appropriate type of prosthesis was selected through the traditional two-dimensional template. Preoperative CT scans of the pelvis and proximal femur were obtained (Siemens, 120 kV, 350 mA, layer spacing < 1 mm). CT data was imported into the Mimics 20.0 software (Master, Belgium). Separate models of the pelvis, healthy femur, injured femoral head, and proximal shaft were established by threshold difference and manual segmentation (Figure 1). After virtual fracture reduction or mirror healthy model registration, the target femoral head center can be obtained by articular surface fitting (Figure 2).

The article "3D Printed Guides and Preoperative Planning for Uncemented Stem Anteversion Reconstruction during Hip Arthroplasty: A Pilot Study" was retracted in 2024. Reasons: suspected computer-generated content; unreliable results or conclusions; concerns about the data; concerns about the results or conclusions.

Then, the femoral stem prosthesis model was imported into the software. Taking the center of the target femoral head as a reference, surgeon adjusted the posture of the prosthetic stem in the front view, lateral view, and top view. In the top view, the axis of the prosthesis's neck passes through the target center. In the front and lateral view, the axis of the prosthesis stem was coaxial with the centerline of the proximal medullary cavity (Figure 3). In group A, 3D process was performed after surgery. In group B, femoral neck osteotomy guide and stem positioning guide were designed (Figure 4). The guide models were output in STL format, printed with 0.1 mm precision photosensitive medical-grade resin. Guides were sterilized by low-temperature plasma.

### 2.3. Surgical Procedure

The operations were performed by the same group of surgeons. All femoral components were made with cementless devices. After receiving general anesthesia or nerve block anesthesia, patients were positioned in the lateral decubitus position for all procedures. The operative technique for both groups was completed using anterolateral approaches. In the group A, surgeons performed operations based on two-dimensional planning and experience. In the group B, 3D preoperative planning was performed before surgery; after exposure of the femoral neck, the bone was cleaned to ensure a secure fit for the guides. Next, the guide was placed in a position to fit around bone in a “best fit” position. The femoral neck osteotomy was performed according to the edge of the guide (Figure 5(b)). After removing the femoral head, the acetabulum was cleaned. Then, the femoral medullary cavity was formed, and the position guide was placed on the osteotomy surface during the forming process (Figure 5(c)). After the stability testing, the femoral steam was implanted according to the guide (Figure 5(d)).

### 2.4. Postoperative Evaluation

All patients received a CT scan prior to discharge using the same technique as the preoperative scans. Evaluation of the final anteversion was determined by superimposing the previous planned stem position to the actual stem position and compared using Tsai's definitions (Figure 6) [3]. From the top view, the planned and postoperative anteversion was measured. The angle difference between the postoperative femoral prosthesis neck axis and the preoperatively planned center was calculated as accuracy value (Figure 6(c)). Cases with the angle change more than 5° were counted as abnormal case.

### 2.5. Statistical Analysis

The data are reported using descriptive statistics, including mean, standard deviation, and range values. The accuracy of the anteversion restoring was compared among groups. Chi-squared test and Mann–Whitney *U* test are used to test differences between groups. *P* < 0.05 was regarded as significant difference.

The article "3D Printed Guides and Preoperative Planning for Uncemented Stem Anteversion Reconstruction during Hip Arthroplasty: A Pilot Study" was retracted in 2024. Reasons: suspected computer-generated content; unreliable results or conclusions; concerns about the data; concerns about the results or conclusions.

## 3. Results

We screened 60 patients and randomized a total of 53 to 2 parallel study arms: 30 patients to the group A (traditional operation) and 23 patients to the group B (3D preoperative planning and 3D printed guide). There were no significant differences in demographic or perioperative data between study groups (Tables 1 and 2).

The average planned anteversion for groups was 22.6° ± 11.4° (group A) and 21.6° ± 9.9° (group B), respectively. The average actual anteversion for groups was 21.8° ± 14.5° and 21.8° ± 10.3°, respectively. The accuracy for groups was 5.42° ± 3.7° (range 0.5° to 17.7°) and 2.32° ± 1.89° (range 0.1° to 6.8°), respectively. The number and rate of abnormal cases was 15 (50%) and 2 (6.7%), respectively. Significant statistical differences were found in angle change, restoration accuracy, and number of abnormal cases.

## 4. Discussion

Component positioning in hip arthroplasty can have a major effect on both clinical outcome and complications rate. Previous studies have focused on the accuracy of acetabular implantation [3, 16–18]. With the introduction of concepts such as combined version, more and more attention has been paid to stem anteversion [19]. Substantial changes in femoral neck version with stem implantation create concurrent changes in anterior and lateral femoral offset, potentially resulting in decrements in abductor strength [20]. Surgical approaches also affect the anteversion change [21].

Traditionally, the recommended positioning for femoral stem is to restore natural offset and anteversion. Various works have in fact shown native femoral neck version that has a wide variation. Abe reported the mean preoperative femoral anteversion was 27.8° ± 10.6° in Japanese population. Koerner reported average femoral version was 8.84° ± 9.66°, with no statistically significant differences between ethnicities [22]. Our study presented similar results that the standard deviation is about 10°. The variable anteversion may cause difficulty for the surgeon to implant correctly.

In order to accurately restore the femoral rotation center, surgeons usually control steam anteversion during the operation, based on experience and visual assessment. But the surgeon's estimation of the anteversion of the cementless femoral stem has poor precision [23]. Wines reported that the mean difference between the surgeons' intraoperative assessment of femoral component version and the CT measurement was an underestimation of 1.18°, with a standard deviation of 10.4° and a range of 25° underestimation to 30° overestimation [24]. In a research of 65 patients, Woerner reported the mean difference between the 3D-CT results and intraoperative estimations by the eye was −7.3° (−34° to 15°) and an overestimation of >5° for stem torsion in 40 hips. Using 3D reconstruction and method, Tsai reported femoral anteversion of the implanted side was significantly increased by 11.4° ± 11.9° [3]. In this study, date of group A also presented that even experienced surgeon's intraoperative estimation of stem position by the eye is not reliable.

The article "3D Printed Guides and Preoperative Planning for Uncemented Stem Anteversion Reconstruction during Hip Arthroplasty: A Pilot Study" was retracted in 2024. Reasons: suspected computer-generated content; unreliable results or conclusions; concerns about the data; concerns about the results or conclusions.

Several studies have investigated the accuracy of measurements obtained using a goniometer or navigation systems [25–27]. Mitsutake developed an angle-measuring instrument; mean measurement accuracy was 0.9° ± 6.1°, and the absolute measurement accuracy was 4.9° ± 3.7° [25]. Using stem-first technique with navigation system, Okada reported absolute discrepancy between intraoperative and postoperative assessment was 5.81° ± 4.42° (range 0.01°–17.4°) [28]. In a robotically assisted study, Marcovigi reported average difference between preoperative and actual stem anteversion was 1.6° ± 9.8° (max 34° in anteversion, min -52° in retroversion). Previous literatures remind that the accurate restoration of femoral anteversion is still a concern for surgeons.

For joint arthroplasty, 3D printed instruments have already been successfully translated into large-scale clinical use for knee arthroplasty. Some studies introduced patient specific instruments that assist acetabular cup placement and femoral neck osteotomy in hip replacements [11, 14]. Lee combined 3D printed instrument and navigation system for an in vitro study with a sawbone model, and the absolute deviation between plan and actual anteversion was 1.41° ± 1.03° (range 0.02°-3.32°) [29]. However, Lee prepared the proximal medullary canal using only a box chisel. Various authors have pointed out that, especially in cementless arthroplasty, the stem finds its way to an anteversion position, where it fits best to the rigid canal of the femur. It should be noted that the entry point of the medullary cavity will affect the anteversion angle and the center of rotation.

For the first time, this article compared the accuracy of anteversion restoration between 3D printed guide and traditional operation. The method of mirror model and virtual reduction was used to determine the target rotation center; then, the personalized osteotomy/positioning guides were designed and manufactured. The results shown that the error of the traditional experience operation is relatively high. The number of abnormal cases is 15 (50%), which is like previous studies. The 3D printed guides improve the accuracy, even better than some navigation system in previous reports. The abnormal case was reduced from 50% to 6.7%. The reason may be that the positioning guide in this experiment is very close to the box chisel and stem, which helps the surgeon choose the appropriate entry point and be a reference during the medullary cavity formation process. The planned stem axis should be overlapped with the proximal medullary cavity axis, which can reduce the mismatch of medullary cavity. In this experiment, the guide does not need to be fixed on the bone and change the surgical procedure slightly.

The article "3D Printed Guides and Preoperative Planning for Uncemented Stem Anteversion Reconstruction during Hip Arthroplasty: A Pilot Study" was retracted in 2024. Reasons: suspected computer-generated content; unreliable results or conclusions; concerns about the data; concerns about the results or conclusions.

## 5. Conclusions

We have proposed the method including 3D planning and 3D printed osteotomy/positioning guides for femoral anteversion restoration. The proposed method was more accurate and consistent than the conventional method. 3D printed guides can reduce the number of inappropriate anteversion. Paying attention to the relationship between the entry point of the box-chisel and the geometry of the osteotomy surface can improve the accuracy of the operation.

## Figures and Tables

**Figure 1:** Fracture modeling build an independent three-dimensional model of fracture through CT.

**Figure 2:** Mirror/virtual fracture reduction, fitting articular surface to determine the target rotation center: front view (a); side view (b); the red circle is the fitting sphere, and the green dot is the planned center.

**Figure 3:** Simulated placement of femoral prosthesis: front view (a), lateral view (b), and top view (c).

**Figure 4:** Design of femoral neck osteotomy guide (a) and prosthesis positioning guide (b).

**Figure 5:** Guide plate printing (a), intraoperative osteotomy (b), intraoperative medullary cavity formation (c), and intraoperative implantation of femoral stem (d).

**Figure 6:** Postoperative modeling and registration (a). Fit the postoperative rotation center (b). Calculate the preoperative planning, the actual postoperative anteversion angle, and the difference (c). Red sphere indicates the planned center; blue sphere indicates the actual center.

**Table 1:** Patient characteristic data.

Variable	Group A	Group B	*P* value
Age at operation (years)	75.5 (54-89)	73.5 (52-86)	0.886^a^
Sex distribution (M/F)	10/20	8/15	0.912^b^
Height (m)	1.61 ± 0.08	1.61 ± 0.08	0.921^a^
Weight (kg)	56.82 ± 10.26	60.48 ± 9.07	0.239^a^
BMI (kg/m^2^)	21.88 ± 3.23	23.34 ± 2.70	0.116^a^
Location (L/R)	17/13	15/8	0.528^b^
Operation type (T/H)	17/13	17/6	0.194^b^

M: male; F: female; L: left hip; R: right hip; BMI: body mass index; T: total hip arthroplasty; H: hemiarthroplasty. ^a^Mann–Whitney *U* test. ^b^Chi-squared test, significance set at *P* < 0.05.

The article "3D Printed Guides and Preoperative Planning for Uncemented Stem Anteversion Reconstruction during Hip Arthroplasty: A Pilot Study" was retracted in 2024. Reasons: suspected computer-generated content; unreliable results or conclusions; concerns about the data; concerns about the results or conclusions.

**Table 2:** Comparison of preoperative and postoperative anteversion.

Variable	Group A	Group B	*P* value
Preoperative femoral anteversion (degrees)	22.61 ± 11.43	21.61 ± 9.96	0.816^a^
Postoperative femoral anteversion (degrees)	21.77 ± 14.48	21.84 ± 10.25	0.971^a^
Anteversion change (degrees)	5.42 ± 3.65	2.32 ± 1.89	0.000^a^
Abnormal case (>5°)	15 (50%)	2 (8.7%)	0.002^b^

^a^Mann–Whitney *U* test. ^b^Chi-squared test, significance set at *P* < 0.05.

## Data Availability

All the data could be provided if any qualified authors required.
